# MRI and DC/TMD Methods Analyze the Diagnostic Accuracy of the Change in Articular Disc of Temporomandibular Joint

**DOI:** 10.1155/2022/1770810

**Published:** 2022-02-15

**Authors:** Shan Shen, Mingjun Ye, Mingle Wu, Wencheng Zhou, Sanghui Xu

**Affiliations:** ^1^Stomatology, The First Affiliated Hospital of Jinan University, Guangzhou 510632, China; ^2^Stomatology, Jinan University Daliang Hospital, Foshan 528300, China; ^3^School of Stomatology, Jinan University, Guangzhou 510632, China

## Abstract

**Methods:**

DC/TMD clinical questionnaire diagnosis was conducted for 30 patients with temporomandibular disorder (TMD) and 11 asymptomatic volunteers who were admitted to the Department of Oral Medicine of the First Hospital affiliated with Jinan University from June 2020 to June 2021. At the same time, MRI scanned the opening and closed positions to obtain the image information of the articular disc and compared the diagnostic difference between MRI and DC/TMD to the position of the articular disc through statistical analysis.

**Results:**

The probability of DC/TMD's diagnosis of reusable/nonreusable anterior disc displacement (ADD) was 80.1% and 62.7%, respectively.

**Conclusion:**

DC/TMD's diagnosis of abnormal articular disc position is less accurate than MRI testing. Therefore, the diagnosis of these two diseases for DC/TMD examination is of little significance, and MRI examination is required at the same time. It can improve diagnosis specificity and sensitivity, reduce missed diagnosis and misdiagnosis rates to ensure that true positive patients can be detected in time, and establish a basis for clinical diagnosis and treatment.

## 1. Introduction

Temporomandibular disorder (TMD) is common in young adults aged 20 to 40 with a prevalence rate of 28% to 88%, mostly in women [1, 2]. In addition, 16%-68% of adolescents also showed symptoms of TMD [3]. Anterior disc displacement (ADD) is one of the most common types of TMD, which is often divided into anterior disc displacement with reduction (DDwR) and anterior disc displacement without reduction (DDwoR) [4]. The displacement and morphological changes between the articular disc and condyle are considered to be important features of the internal disorder of the joint and a cause of dysfunction.

MRI, as an imaging diagnostic method that can show the TMJ, is considered to be the gold standard of the current TMD examination, which can diagnose the change of the anterior disc position [5, 6]. Currently, commonly used MRI checks include open and closed oblique vector T1WI, T2WI, PDWI scanning, and oblique coronal PDWI scanning. Studies have shown that people without symptoms of joint discomfort find abnormalities such as changes in the position of the anterior disc when they perform ANI scans in recent years [7]. Whether or not such people are diagnosed with TMD is uncertain. In this study, the difference between MRI and DC/TMD's diagnosis of anterior disc position is discussed by analyzing the MRI of DC/TMD results. At present, TMD patients are diagnosed with more obvious symptoms by the TMD Diagnostic Standard (DC/TMD). However, whether this diagnostic model can give clinicians enough information and guide the correct diagnosis and treatment plan is still controversial.

## 2. Information and Methods

### 2.1. Information

Patients admitted to the First Hospital affiliated with Jinan University between June 2020 and February 2021 were divided into the TMD group (30 cases) and the control group without temporomandibular joint (TMJ) symptoms and pain (11 cases). Magnetic resonance imaging (MRI) is performed to obtain the regular sequence of MRI after initial diagnosis by DC-TMD assessment/diagnosis questionnaire. 38 people aged 17-56 years were screened, of whom 11 were men and 27 were women with an average age of 26 years. Patients were divided into 3 groups according to the preliminary diagnosis results of the DC/TMD clinical questionnaire: normal group (NL group, 21 cases), DDwR group (14 cases), and DDwoR group (19 cases). The patients were divided into 3 groups by the results of the MRI scan: M-NL group (47 cases), M-DDwR group (9 cases), and M-DDwoR group (20 cases).

### 2.2. Inclusion and Exclusion of Standards

Inclusion standards of the TMJ group are as follows:

(1) The presence of shifters in TMJ is diagnosed strictly following DC/TMD [8]
(2) Inclusion standards of TMJ without symptom and pain
  - Without the history of pain in the anterior disc or other craniomaxillofacial pain disease was diagnosed according to DC/TMD [9]. All volunteers read and signed the patient informed book, which described the study in detail
(3) Exclusion criteria of all subjects
  - Gestation period
  - A history of neurological or mental illness
  - History of oral and maxillofacial trauma and/or special medications taken
(4) Systemic diseases such as rheumatism, rheumatoid arthritis, and tumors; other coexisting chronic pain such as fibromyalgia
(5) History of TMD treatment, such as analgesics, physiotherapy, and Lidocain closure
(6) MRI contraindications, such as claustrophobia, in people with pacemakers or metal prosthetics in a person's body

### 2.3. Check Method

Each study subject and volunteer was required to fill out basic information and DC/TMD tables to count clinical symptoms and other information before scanning. Patients or volunteers are examined before scanning to ensure that there are no MRI contraindications. All metal magnetic items were removed from the body, and earplugs were worn to reduce noise to protect the patient's hearing before performing an MRI. The patient's head was secured with a sponge, the patient was instructed to lie on his back on the scan bed, and the patient was told to remain still during the scan.

The scanner is a Signa GE HDxt 1.5 T scan with superconducting MRI scanner, and the scanning coil is a DUAL TMJ coil. The patient takes the resting position (body in center, head in advance). Two sides of the mandibular condyle are located in the center of the coil; the center of the coil is placed in the center of the magnet to ensure that the two-sided mandibular condyle connection center, coil center, and magnet center are located in the same center. The precise anatomical structure and its positional relationship are obtained by T1WI imaging of the horizontal axle surface perpendicular to the long axis of the mandibular condyle to determine the structure and position of the mandibular condyle. Then, the oblique corona and oblique symography scans are carried out in parallel and perpendicular to the mandibular condyle, respectively. The TMJ scan is preceded by a closed-mouth check (tell the patient to grit his back teeth) and then an open-mouth check (with a plastic opener opening to the comfortable position until it cannot be opened). The scanning method and parameters are the same as the closed-mouth position. The same scanning conditions were completed by the same imaging lead technician. Scan sequences and parameters are shown in Table 1.

*Image evaluation methods and observation indicators*: the scanned images were analyzed and counted by two doctors using double blindness.

MRI image observation indicators for TMJ of TMD patients are as follows:

(1) The articular disc shifts [10]:
  - *Normal*: the rear band of the articular disc is located at a position of 12 o'clock relative to the condylar apex at the closed position. The combination of the rear belt and the double plate area is located within a range of 10 degrees at 12 o'clock. The back belt is in the backside position of 12 o'clock for the normal disc-burst relationship on the opening position (Figure 1).
  - *DDwR*: the back strap of the articular disc moves forward beyond the normal range, and the opening position returns to the normal disc-burst position at the closed position (Figure 2).
  - *DDwoR*: the back strap of the articular disc moves forward beyond the normal range, and the opening position cannot be restored to the normal disc-burst position at the closed position (Figure 3).
(2) Articular disc shape [11]^:^
  - *Normal*: normal articular disc shape (Figures 4(a) and 5(a)).
  - *Folded*: twisted articular disc (Figures 4(b) and 5(b)).
  - *Lengthened*: an articular disc that is longer than the normal length (Figures 4(c) and 5(c)).
  - *Round*: a circular articular disc that loses its concave structure (Figures 4(d) and 5(d)).
  - *Biconvex*: loss of concave shuttle articular disc (Figures 4(e) and 5(e)).
  - *Thick*: an articular disc that thickens according to its normal size (Figures 4(f) and 5(f)).

### 2.4. Statistical Analyses

The experimental data are statistically analyzed using SPSS 27.0 software. Measures that obey normal distributions are expressed in average ± standard deviation$\left(\bar{x}\pm s\right)$. The mean between the two groups was compared using a separate sample *t*-test. The variance analysis is used in the comparison between the groups, and the LSD method is used for correction. Measurements that do not follow the normal distribution are expressed in the median (quartile range) [*M*(*P*_25_, *P*_75_)]. The nonparametric Mann–Whitney *U* test was used for comparison between the two groups, and the correlation between variables was analyzed using Spearman dependencies. Counting data is expressed in frequency (percentage) [*n*(%)].The differences between groups are compared using the *χ*^2^-test and Fisher's exact probability method. *P* < 0.05 is considered statistically significant.

## 3. Results

The diagnosis relationship between DC/TMD and MRI. The diagnosis efficacy of DC/TMD and MRI.

The results are shown in Table 2. The difference between DC/TMD and MRI diagnosis in 27 patients was statistically significant (*P* < 0.05).

The ROC curve is drawn using MRI as the gold standard. Comparison of the position of DC/TMD in the articular disc to change the diagnostic efficacy of disease is shown in Figures 6 and 7. The diagnosis efficacy of DC/TMD is shown in Figures 6 and 7. DC/TMD's diagnosis of DDwR/DDwoR was 80.1% and 62.7%, respectively.

1. DDwR
2. DDwoR

## 4. Discussion

TMD is a common disease of the oral jaw and facial caused by a variety of factors, which is common in middle-aged and young people. However, the rate of visits is only about 10% of the total prevalence [12]. Clinical symptoms of TMD are most common with functional disorders such as joint pain, bite, and limited opening. The etiology and pathogenesis of this disease are not clear. Therefore, accurate classification and diagnosis with TMD is the key and prerequisite for treatment.

DC/TMD is a clinical diagnostic tool that has been widely used in the world. The diagnostic criteria are used as a preliminary judgment through medical history collection and clinical examination without relying on imaging or other auxiliary examinations. TMD patients can receive a “relatively” accurate classification diagnosis according to the classification and diagnostic criteria of DC/TMD [9]. The DC/TMD axis I protocol is not only an effective screening method for any pain-related TMD patient but also a diagnostic criterion for the most common pain-related TMD (sensitivity ≥ 0.86 and specificity ≥ 0.98) and intrajoint disorders (sensitivity ≥ 0.80, specificity ≥ 0.97). Axis II protocol retains the selected original RDC/TMD screening tool and uses new diagnostic tools to evaluate jawbone function as well as motor and other psychosocial factors. It can be used to understand the pain level of patients with TMD and jaw function restriction [13]. Step-by-step systematic examination is done according to the DC/TMD questionnaire, which is conducive for the consolidation of medical records and reduces the chance of missed diagnosis and misdiagnosis. It is more conducive for the analysis of causes and treatment.

The DC/TMD diagnostic method has certain sensitivity and specificity, but there are also problems. It is statistically significant by analysis of the relationship between DC/TMD and MRI diagnosis (*P* < 0.05). The ROC curve analysis showed that the DC/TMD and MRI compliance rate reached 80.1% in the diagnosis of DDwR. However, the diagnostic and MRI compliance rate for DDwoR was only 62.7%, which indicates that DC/TMD diagnosis is not accurate enough. In this study, volunteers who were initially diagnosed as asymptomatic and painless by DC/TMD method found different degrees of disc displacement, articular disc deformation, and bone changes in the joints when they were rediagnosed with MRI imaging. Kumar and Brennan point out that compensation and degenerative changes can occur when an internal disorder in the joint fails to restore biometric balance [14]. Joints may show no or very light symptoms for a period of time due to the joint's ability to adapt, which requires a combination of careful clinical evaluation and imaging examination to assist in diagnosis. TMJ asymptomatic pain-free cannot necessarily be used as a healthy control, and joint disc morphology or location abnormalities may not be able to become the basis for the diagnosis of articular disc lesions. Therefore, this study only takes DC/TMD as a preliminary diagnosis and uses MRI for clear diagnosis and grouping. It also states that the DC/TMD is not sufficient to diagnose TMD and needs to be assisted by imaging examination. In addition, most patients showed one-sided clinical manifestations with no abnormalities on the other side. However, MRI examination can find that the two-sided joints often appear in varying degrees of articular disc shift, fluid, malformation, and bone defects. This indicates that asymptomatic joints may also be lesions. Therefore, DC/TMD clinical manifestations as the main observation indicators of a diagnosis are unable to effectively judge the condition and stage of the joint.

## 5. Conclusion

This helps to establish the basis of clinical diagnosis and treatment by detecting real positive patients in clinical work on time.

## Figures and Tables

**Figure 1:** Normal disc-process position: (a) closed position; (b) opening position.

**Figure 2:** Disc displacement with reduction: (a) closed position; (b) opening position.

**Figure 3:** Disc displacement without reduction: (a) closed position; (b) opening position.

**Figure 4:** Articular disc shape: (a) normal; (b) folded; (c) lengthened; (d) round; (e) biconvex; (f) thick.

**Figure 5:** Articular disc shape: (a) normal; (b) folded; (c) lengthened; (d) round; (e) biconvex; (f) thick.

**Figure 6:** Diagnostic efficacy of DDwR in DC/TMD.

**Figure 7:** Diagnostic efficacy of DDwoR in DC/TMD.

**Table 1:** 1.5 T MRI of the general sequence and parameters of TMJ.

Project	Horizon (mm)	Thickness (mm)	Layer spacing (mm)	Repetition time (ms)	Echo time (ms)	Number of excitations	Acquisition matrix (mm)
T1WI (sagittal plane)	120 × 120	2	0.2	400	12	4	256 × 224
T2WI fs (sagittal plane, fat suppression)	120 × 120	2	0.2	3000	85	4	256 × 224
T2WI PDWI (coronal axial plane)	120 × 120	2	0.2	3000	40	4	256 × 224
T1WI (coronal axial plane)	120 × 120	2	0.2	400	12	4	256 × 224

**Table 2:** Relationship between DC/TMD diagnosis and MRI diagnosis.

Group	Subgroups	MRI diagnosis (*N*, %)			*P* value
		Normal group	M-DDwR group	M-DDwoR group	
DC/TMD diagnosis	Normal group	15 (57.7)	3 (33.3)	3 (15.8)	0.003^∗∗^
	DDwR group	7 (26.9)	4 (44.4)	3 (15.8)	
	DDwoR group	4 (15.4)	2 (22.2)	13 (68.4)	
Total		26 (100.0)	9 (100.0)	19 (100.0)	

## Data Availability

No data were used to support this study.

## References

[1] Cui J., Zhang X. Y., Zhang Z. L. (2018). Advances in the study of psychological conditions in patients with temporomandibular disorder. *Chinese Journal of Geriatric Dentistry*.

[2] Wu M., Zhang J. (2020). Research progress on acupuncture and massage treatment of temporomandibular joint disorders. *China Journal Medicial Guide*.

[3] Chang C. L., Wang D. H., Yang M. C., Hsu W. E., Hsu M. L. (2018). Functional disorders of the temporomandibular joints: internal derangement of the temporomandibular joint. *Medical Science*.

[4] Zhang Q., Li J., Ma L. X., Wang Z. H. (2021). Diagnostic value of temporomandibular joint open and closed magnetic resonance imaging in anterior disc displacement of temporomandibular joint. *Journal of Imaging Research and Medical Applications*.

[5] Tasaki M. M., Westesson P. L., Isberg A. M., Ren Y. F., Tallents R. H. (1996). Classification and prevalence of temporomandibular joint disk displacement in patients and symptom-free volunteers. *American Journal of Orthodontics and Dentofacial Orthopedics*.

[6] Koh K. J., Park H. N., Kim K. A. (2013). Relationship between anterior disc displacement with/without reduction and effusion in temporomandibular disorder patients using magnetic resonance imaging. *Imaging Science in Dentistry*.

[7] Larheim T. A. (2005). Role of magnetic resonance imaging in the clinical diagnosis of the temporomandibular joint. *Cells, Tissues, Organs*.

[8] Wänman A., Marklund S. (2020). Treatment outcome of supervised exercise, home exercise and bite splint therapy, respectively, in patients with symptomatic disc displacement with reduction: a randomised clinical trial. *Journal of Oral Rehabilitation*.

[9] International RDC/TMD Consortium Network (2014). Diagnostic criteria for temporomandibular disorders (DC/TMD) for clinical and research applications: recommendations of the international RDC/TMD consortium network and orofacial pain special interest group. *Journal of Oral & Facial Pain and Headache*.

[10] Meluzinová P., Kopp L., Dráč P., Edelmann K., Obruba P. (2017). Comparison of short-therm results of conservative versus operative treatment of distal ulna fractures associated with distal radius fracture treated by plate osteosynthesis. *Acta Chirurgiae Orthopaedicae et Traumatologiae Cechoslovaca*.

[11] Murakami T., Otsuki S., Nakagawa K. (2017). Establishment of novel meniscal scaffold structures using polyglycolic and poly-l-lactic acids. *Journal of Biomaterials Applications*.

[12] Slade G. D., Sanders A. E., Bair E. (2013). Preclinical episodes of orofacial pain symptoms and their association with health care behaviors in the OPPERA prospective cohort study. *Pain*.

[13] Schiffman E., Ohrbach R. (2016). Executive summary of the diagnostic criteria for temporomandibular disorders for clinical and research applications. *Journal of the American Dental Association*.

[14] Kumar A., Brennan M. T. (2013). Differential diagnosis of orofacial pain and temporomandibular disorder. *Dental Clinics of North America*.

